# Risk Factors and Nursing Countermeasures of Ventilator-Associated Pneumonia in Children in the Intensive Care Unit

**DOI:** 10.1155/2022/9055587

**Published:** 2022-02-17

**Authors:** Rong Chen, Yu Liu, Xiaohong Zhang, Qin Yang, Xiao Wang

**Affiliations:** Department of ICU, Xiangyang Central Hospital, Affiliated Hospital of Hubei University of Arts and Science, Xiangyang, Hubei 441021, China

## Abstract

**Objective:**

This study discussed and analyzed the risk factors and nursing countermeasures of ventilator-associated pneumonia (VAP) in the children intensive care unit (ICU).

**Methods:**

In this study, 155 children with mechanical ventilation in the pediatric intensive care unit from Oct. 2018 to Oct. 2020 were chosen as research objects. We retrospectively analyzed the clinical data of children and divided them into VAP groups and non-VAP groups according to the occurrence of VAP. Subsequently, we adopted a univariate and multivariate logistic regression model to analyze and clarify the risk factors of VAP and formulated the corresponding nursing countermeasures.

**Results:**

49 cases of total research objects had occurred VAP, with an infection rate of 31.62%. The primary pathogenic bacteria were Gram-negative bacteria (43/70, 61.43%). According to multivariate logistic regression analysis, the duration of mechanical ventilation, invasive procedures, and application of hormones and antacids are all independent risk factors for VAP in pediatric ICU. The VPA group had longer hospital stay than the non-VAP group, and the difference was statistically significant ((20.92 ± 4.16)d, (15.24 ± 3.77)d, *t* = 8.4383, *P* ≤ 0.001). The hospitalization cost of the VPA group was substantially higher than that of the non-VAP Group ((45.8 ± 10.4) thousand Yuan, (33.2 ± 4.3) thousand Yuan, *t* = 10.6822, *P* ≤ 0.001).

**Conclusion:**

Children admitted to the pediatric ICU have a high VAP incidence. The primary pathogenic bacteria are Gram-negative bacteria. As the occurrence of VAP is closely related to a variety of factors, we should take targeted nursing countermeasures to reduce the duration of mechanical ventilation and the frequency of invasive operations and use the hormone and antacids rationally to reduce the risk of VAP and improve the prognosis.

## 1. Introduction

Most children admitted to the pediatric intensive care unit (ICU) have severe pneumonia, myocarditis, encephalitis, hand-foot-and-mouth disease, etc. Children often need to use respiratory support to get through the dangerous period due to respiratory disorders or respiratory failure, but the application of ventilator is easy to cause complications such as pulmonary injury, displacement of tracheal intubation, septic shock, and respiratory-associated pneumonia (VAP) [1, 2]. VAP refers to pulmonary infection that occurs 48 h after endotracheal intubation or tracheostomy with mechanical ventilation or 48 h after removal of a mechanical ventilation tube, which has high morbidity and fatality rate [3, 4]. VAP prolongs the length of hospital stay and surcharges medical costs and increases the clinical mortality rate and affects the prognosis of children [5]. In recent years, the risk factors of VAP have been the hot spot in the analysis and research of the intensive care field. According to the work in [6–8], the occurrence of VAP is closely related to clinical nursing operations. Therefore, it is of great significance to take effective preventive and nursing measures to reduce VAP risks in the pediatric ICU. This study retrospectively analyzed the clinical data of the 155 mechanically ventilated children in the pediatric ICU of our hospital from Oct. 2018 to Oct. 2020, aiming to clarify the risk factors, pathogen distribution characteristics, and prognosis of children admitted in our pediatric ICU with VAP, meanwhile, to find targeted nursing countermeasures for the pediatric ICU of our hospital, and to provide a theoretical basis for clinical prevention of VAP.

## 2. Cases and Methods

### 2.1. General Data

155 children with mechanical ventilation in the pediatric ICU from Oct. 2018 to Oct. 2020 were chosen as research objects. The objects included 81 males and 74 females, with an average age of (7.83 ± 2.46) years; the average duration of mechanical ventilation was (7.35 ± 3.12)d, and the average length of hospital stay was (18.52 ± 3.05)d. This study was carried out after acquiring approval from the ethics committee of our hospital.

### 2.2. Inclusion and Exclusion Criteria

Inclusion criteria: (1) the age of the patients ranged from 3 to 12 years; (2) all children were treated with invasive ventilation, and the duration of mechanical ventilation was ≥48 d; (3) children tended to be in stable conditions, or without progressive aggravation; and (4) the clinical data of children were complete.

Exclusion criteria: (1) children that were diagnosed with severe pneumonia before mechanical ventilation; (2) children with other serious diseases; (3) children with conscious or cognitive disorders, or with mental disorders; or (4) those discharged or died during treatment.

### 2.3. Diagnostic Criteria of VAP

We performed chest X-ray examination on children who have received mechanical ventilation for 48 h or within 48 h of withdrawing the ventilator and intubation. X-ray shows infiltrative shadows or new inflammatory lesions in the lungs, and moist rales could be heard during auscultation. According to the diagnostic criteria of VAP in *Guidelines for the Diagnosis and Treatment of Hospital-Acquired Pneumonia of the Chinese Society of Respiratory Medicine* [9], the child met any of the following two conditions simultaneously: (1) body temperature >38.5°C or <36.5°C, and there were no other obvious external causes; (2) the white blood cell (WBC) >10 × 10^9^/L or <4.0 × 10^9^/L; (3) increased or purulent respiratory secretions; and (4) new pathogenic bacteria were cultured in secretions.

### 2.4. Methods

We took 155 children with mechanical ventilation in the pediatric intensive care unit from Oct. 2018 to Oct. 2020 as research objects, retrospectively analyzed their clinical data, and divided them into VAP groups and non-VAP groups according to VAP occurrence. The children's general clinical data include gender, age, underlying diseases, blood transfusion experience, nutritional status, diagnosis, and treatment conditions such as nutritional support methods, intubation methods, application of antibiotics and hormones, and duration of mechanical ventilation retrospectively analyzed. We performed a single-factor analysis on the respective risk factors of the two groups and subsequently incorporated the obtained high-risk factors into the logistic regression model for analysis.

### 2.5. Statistical Analysis

We adopted the statistical software SPSS19.0 to analyze and process the data included. The measurement data were expressed as ($\bar{x}$ ± s), and comparison between groups was by the *t*-test of independent samples; the enumeration data were described by percentage, and the results were taken by *χ*^2^. *P* < 0.05 refers to the statistically significant difference. The multivariate logistic regression analysis included the selected statistically significant variables to determine independent risk factors by steps, and the significance level *α* = 0.05.

## 3. Results

### 3.1. General Clinical Data in the Pediatric ICU

49 cases of real research objects had occurred VAP, the infection rate was 31.62%, and a total of 70 pathogens were detected (Table 1). According to univariate analysis, the general clinical data of patients, including age, underlying diseases, experience of blood transfusion, and malnutrition, were all connected with the occurrence of VAP (Table 2).

### 3.2. Univariate Analysis of Medication and Diagnosis

Univariate analysis results indicated that the diagnosis and treatment, such as duration of mechanical ventilation, length of ICU stay, and application of invasive operations and hormones and antibiotics, were all concerned with the occurrence of VAP, as shown in Table 3. Variable assignment of VAP in the pediatric ICU: the variable assignment of VAP in the child intensive care unit is shown in Table 4. According to multivariate logistic regression analysis, the duration of mechanical ventilation, invasive procedures, and application of hormones and antacids are all independent risk factors for VAP in the pediatric ICU (Table 5).

### 3.3. Comparison of Treatment between the Two Groups of Children in the ICU

The VPA group had longer hospital stay than the non-VAP group, and the difference was statistically significant ((20.92 ± 4.16)d, (15.24 ± 3.77)d, *t* = 8.4383, *P* ≤ 0.001); the hospitalization cost of the VPA group was substantially higher than that of the non-VAP group [(44.58 ± 1.04) ten thousand Yuan, (3.32 ± 0.43) ten thousand Yuan, *t* = 10.6822, *P* ≤ 0.001) (Table 6 and Figure 1).

## 4. Discussion

Mechanical ventilation is a treatment that applies a ventilator to alter or replace patient's active breathing. It relies on auxiliary equipment to establish the pressure difference between the airway orifice and the alveoli of patient, thus alleviating the respiratory failure or dyspnea of the patient [10, 11]. According to the literature, over 20% children in the pediatric ICU will be treated with mechanical ventilation during treatment [12]. The complication of VAP in children often occurs with the widespread application of mechanical ventilation in the pediatric ICU. For every 24 h increase in time of mechanical ventilation, the probability of VAP will increase by 1% to 3%. According to related data [13], the incidence rate of VAP in children with mechanical ventilation was 9%–68%, the mortality was 24%–76%, and the incidence tends to increase year by year. Through the investigation of pathogenic bacteria changes in VAP children, it has been found in related studies that the primary pathogenic bacteria of VAP are Gram-negative bacteria, which have multiple drug resistance [14]. The primary pathogens of VAP in the pediatric ICU, of our hospital during the past 2 years, are *Acinetobacter baumannii*, *Staphylococcus aureus*, *Klebsiella pneumoniae*, and *Pseudomonas aeruginosa*. These results are consistent with those of most research [15–17].

The results of this study's univariate analysis and multivariate logistic regression analysis showed that the duration of mechanical ventilation, invasive operations, and the application of hormones and antacids are all independent risk factors for VAP in the pediatric ICU. The duration of mechanical ventilation is positively correlated with VAP incidence, and the incidence of VAP increases with the extension of mechanical ventilation. This is because the immunity of children under the growing and developing stage is weak due to incomplete body development. During mechanical ventilation, the normal physiological barriers of the nose, throat, and tracheal mucosa of the child are vulnerable to being damaged, which reduces the movement capacity of cilia and increases the viscosity of sputum, as well as chances pathogen invasion and reproduction, thus leading to the occurrence of nosocomial infection [18, 19]. The long-term mechanical ventilation also aggravates lung injury. The long-term upper respiratory tract stimulation of patients increases the accumulation of sputum and oesophagal reflux in children, which increases the probability of pathogens entering the lung tissues and terminal bronchi, thereby further increasing the risk of VAP [20]. Children with invasive operations are prone to VAP, which may be related to the aspiration and regurgitation of colonizing bacteria, the contamination of mechanical ventilation pipes, and the improper operations of medical staff [21, 22]. Glucocorticoids have effects of anti-inflammatory, antiviral, antishock, and immune suppression, but the inappropriate use will reduce the body defence function of children and interfere with electrolyte balance and energy metabolism in the body. This will increase bacterial infection in children and lead to bacterial resistance, resulting in adverse outcomes such as severe pneumonia and immunodeficiency [23, 24] and rising VAP incidence in the pediatric ICU. The use of antacids increases VAP incidence, and its dominant reason may be that antacids can increase the PH value of gastric juice, thus weakening the gastric acid barrier in children. This can lead to gastrointestinal dysbacteriosis in children, leading to infections with multidrug-resistant bacteria such as *Acinetobacter baumannii* and *Klebsiella pneumonia*. On the other hand, the increased application of antacids may also lead to the displacement of the intestinal flora of children or the migration of colonizing bacteria to the lungs caused by oesophagal reflux, thus increasing VAP's probability [25, 26].

Given the independent risk factors for the occurrence of VAP in the pediatric ICU, our hospital has organized and formed the following targeted nursing countermeasures based on routine care. (1) Strengthening the humidification management of artificial airways and adjusting the total amount of humidification in line with the children's disease stouts and the viscosity of sputum. Appropriate airbag inflating pressure should be used, an adequate airtight artificial airway should be formed, the probability of external bacteria entering the respiratory tract should be reduced, and the respiratory infections caused by hand contamination should be prevented; subglottic sputum aspiration should be used, which can effectively clear the sputum and reduce the probability of pulmonary disease; intermittent shutdowns should be taken, the changes in the children's vital signs should be closely monitored, the intubation and ventilator should be removed as soon as possible to reduce the treatment time of mechanical ventilation, and the recovery of children's spontaneous breathing should be promoted [27, 28]. (2) The aseptic operations should be strictly followed when performing invasive operations. The pipeline should be checked immediately after operation to confirm whether it is polluted, the nursing should be strengthened, and the channel should be disinfected in time to prevent the reproduction of colonizing bacteria, thereby reducing the risk of VAP in children. (3) The sensitive drugs should be selected following the detection results of pathogenic bacteria in children, the changes and drug resistance of infected strains should be monitored by the dynamic method, and timely adjustments should be made to the types, duration, and dosage of hormones. (4) Gastric mucosal protectants instead of antacids should be used according to the child's condition to prevent gastrointestinal bleeding; dietary guidance and oral care should be strengthened. According to studies, the nursing countermeasures can remarkably reduce the incidence of VAP and prevent secondary infection, which is an effective measure to improve the patient's quality of life [29, 30].

## 5. Conclusions

To conclude, children admitted to the pediatric ICU have a high VAP incidence; the primary pathogenic bacteria are Gram-negative bacteria. As the occurrence of VAP is closely related to a variety of factors, we should take targeted nursing countermeasures to reduce the duration of mechanical ventilation and the frequency of invasive operations and use the hormone and antacids rationally to reduce the risk of VAP and improve the prognosis.

## Figures and Tables

**Figure 1:** Comparison of the treatment of children in the ICU between the two groups. Compared with the non-VAP group, ^*∗*^*P* < 0.05.

**Table 1:** Distribution of pathogenic bacteria of VAP in the pediatric ICU.

Species of pathogenic bacteria	Quantity	Composition ratio (%)
Gram-negative bacteria	43	61.43
*Acinetobacter baumannii*	19	27.14
*Klebsiella pneumoniae*	8	11.43
*Pseudomonas aeruginosa*	8	11.43
*Stenotrophomonas maltophilia*	4	5.71
*Escherichia coli*	3	4.29
*Enterobacter cloacae*	1	1.43
Gram-positive bacteria	23	32.86
*Staphylococcus aureus*	15	21.43
*Staphylococcus epidermidis*	5	7.14
*Enterococcus*	3	4.29
Fungi	4	5.71
*Candida albicans*	4	5.71
Total	70	100

**Table 2:** Univariate analysis of general clinical data on VAP in the pediatric ICU.

General clinical data	VAP group (*n* = 49)	Non-VAP group (*n* = 106)	*X* ^2^	*P*
Gender (cases)			0.0185	0.8918
Male	26	55		
Female	23	51		
Age (yd)			11.9029	0.0006
<7	28	30		
≥7	21	76		
Underlying disease (cases)			12.2373	0.0005
Yes	26	26		
No	23	80		
Experience of blood transfusion (case)			12.4831	0.0004
Yes	25	24		
No	24	82		
Malnutrition (cases)			5.7306	0.0167
Yes	13	12		
No	36	94		

**Table 3:** Univariate analysis of VAP diagnosis and treatment in the pediatric ICU.

Factors of diagnosis, treatment, and medication	VAP group (*n* = 49)	Non-VAP group (*n* = 106)	*X* ^2^	*P*
Methods of nutritional support (cases)			2.7389	0.0979
Parenteral nutrition	35	61		
Enteral nutrition	14	45		
Intubation method (cases)			1.2000	0.2733
Mouth	25	64		
Transnasal	24	42		
Duration of mechanical ventilation (cases)			10.9749	0.0009
<7 d	17	67		
≥7 d	32	39		
Duration of stay in the ICU (cases)			6.9206	0.0085
<48 h	18	63		
≥48 h	31	43		
Invasive operations (cases)				
Yes	38	53	10.4927	0.0012
No	11	53		
Application of antibiotics (cases)			0.8126	0.3674
Exclusive use	26	48		
Jointly use	23	58		
Application of hormone (cases)			22.0874	0.001
Yes	36	35		
No	13	71		
Application of antibiotics (cases)			20.8232	0.001
Yes	22	86		
No	27	20		
Atomizing inhalation (cases)			2.8590	0.0909
Yes	19	63		
No	30	43		

**Table 4:** Variable assignment of VAP.

Variables	Explanation of assignment
Age	<7yd = 1, ≥7 = 0
Underlying diseases	YES = 1, NO = 0
Experience of blood transfusion	YES = 1, NO = 0
Malnutrition	YES = 1, NO = 0
Duration of mechanical ventilation	≥7 d = 1, <7 d = 0
Time of admission to the ICU	≥48 h = 1, <48 h = 0
Invasive operations	YES = 1, NO = 0
Use of hormones	YES = 1, NO = 0
Application of antibiotics	YES = 1, NO = 0

**Table 5:** Multivariate logistic regression analysis of VAP in the pediatric ICU.

Factor	*β*	S. E	Wald *X*^2^	*P*	OR	95% CI
Mechanical ventilation	1.232	0.421	8.564	0.003	3.428	1.502–7.824
Invasive operations	1.496	0.425	12.390	≤0.001	4.464	1.941–10.286
Application of hormones	2.137	0.736	8.431	0.004	8.474	2.003–35.858
Application of antacids	1.535	0.524	8.581	0.003	4.641	1.662–12.962

**Table 6:** Comparison of the treatment of children in the ICU between the two groups.

Group	Length of hospital stay (d)	Hospital expenses (ten thousand Yuan)
VAP group (*n* = 49)	20.92 ± 4.16	4.58 ± 1.04
Non-VAP group (*n* = 106)	15.24 ± 3.77	3.32 ± 0.43
T	8.4383	10.6822
*P*	0.001	0.001

## Data Availability

The data used to support this study are available from the corresponding author upon request.
